The article "Risk Factors of Benign Stricture of Anastomotic Stoma after Esophagectomy and Therapeutic Effect of Stent Implantation" was retracted in 2024. Reasons: signs of a paper mill; suspected computer-generated content; unreliable results or conclusions; lack of ethics approval or compliance.

# Risk Factors of Benign Stricture of Anastomotic Stoma after Esophagectomy and Therapeutic Effect of Stent Implantation

**DOI:** 10.1155/2022/2605592

**Published:** 2022-08-30

**Authors:** Guoliang Wu, Lihua Niu, Yanlin Yang, Shaoyong Tian, Yanru Liu, Chunyan Wang, Pengfei Zhao

**Affiliations:** ^1^Department of Interventional Radiology, Harrison International Peace Hospital, Hengshui, Hebei 053000, China; ^2^Department of Ultrasound, Hengshui Chinese Medicine Hospital, Hengshui, Hebei 053000, China; ^3^Department of Culture and Education, Hengshui Health School, Hengshui, Hebei 053000, China; ^4^Department of Radiology, Hengshui Chinese Medicine Hospital, Hengshui, Hebei 053000, China

## Abstract

With the increase in the number of patients and prolongation of their lives after esophagectomy for esophageal cancer, the quality of life after surgery has attracted more and more attention. Although anastomotic stenosis is a common complication, it seriously affects the quality of life and psychological state of patients or even threatens their lives. At present, the exact independent influencing factors of anastomotic stenosis after esophageal cancer surgery have not been determined, and relevant treatment options are still controversial. Here, we analyzed the independent risk factors leading to good postoperative anastomotic stenosis, in order to provide a basis for late prevention. At the same time, we deeply discussed the advantages and safety of stent implantation in the treatment of anastomotic stenosis.

## 1. Introduction

Esophageal cancer is a common clinical malignant tumor, and its incidence is second only to gastric cancer [1]. According to an epidemiological survey, the mortality rate of this disease accounts for 20% of all malignant tumors [2]. Therefore, surgical treatment should be carried out as soon as possible. Although the curative effect has been affirmed with the introduction of minimally invasive surgery, postoperative complications have remained high, including gastric emptying disorders, reflux esophagitis, chylothorax, and anastomotic stenosis[3]. Among them, anastomotic stenosis is the most common, with an incidence rate as high as 15.2%–42.7% [4]. At the same time, postoperative esophageal anastomotic stenosis can lead to pain, difficulty, vomiting, food regurgitation, and even malnutrition in severe cases, requiring reoperation [5]. If it is not prevented and treated in time, it can have a serious impact on the prognosis. Therefore, the factors of postoperative stenosis should be included in the key observation objects. Although scholars have explored the prognostic factors after esophageal cancer surgery, there are few related reports, and the exact independent influencing factors have not yet been determined [6]. The basis for later prevention is provided, and the advantages and safety of stent implantation in anastomotic stenosis are further analyzed. The report is as follows.

## 2. Materials and Methods

### 2.1. General Information

From February 2018 to December 2021, 92 patients with esophageal cancer surgery were selected as the research subjects. There were 51 males and 41 females, with an average age of 58.65 ± 6.65 years, and an average tumor diameter of 2.31 ± 0.75 cm; TNM stage: 32 cases of stages I∼II and 60 cases of stages III∼IV. The study was complied with the Declaration of Helsinki for ethical review. According to the presence or absence of benign anastomotic stenosis after the operation, the patients were divided into two groups, namely, the stenosis group (grades I, II, and III; *n* = 55) and the nonstenosis group (grade 0; *n* = 37).

### 2.2. Inclusion Criteria

Inclusion criteria were as follows: ① All patients who met the diagnostic criteria for esophageal cancer and underwent surgical treatment [7]. The stenosis group also needed to meet the diagnostic criteria of benign stenosis of the anastomosis, the specific criteria are as follows: grade IV: severe stenosis, cannot be expanded, and needs to be relieved by surgery; grade III: three or more consecutive dilations are required and repeated esophageal strictures; grade II: dilation ≤2 times, anastomotic diameter <1 cm, and eating semiliquid disorder; grade I: slight obstruction to eating, no need for expansion; and grade 0: there is no stricture of the anastomotic stoma, and there is no obstruction to eating [8]. ② Patients whose postoperative survival time was more than 6 months. ③ Patients whose esophagus-stomach anastomosis was used in all operations and the esophagus was reconstructed by the tubular stomach. ④ Patients whose clinical data were complete were included in this study.

### 2.3. Exclusion Criteria

Exclusion criteria were as follows: ① patients with 2 or more malignant tumors, ② patients with total pharyngeal esophagectomy, and ③ patients with external esophageal pressure, achalasia, hiatal hernia, and neurogenic dysphagia.

### 2.4. Data Survey

The general data of the patients were evaluated using a questionnaire developed by the hospital, including age, gender, anastomosis method, tumor diameter, pathological type, past medical history, TNM stage, expansion method, anastomotic stoma location, local blood supply, and eating time.

### 2.5. Therapeutic Method

0.5 mg of atropine and 10 mg of diazepam were intramuscularly injected 30 minutes before surgery, and 10 mL of lidocaine mucilage was orally administered. Taking the left lateral position, we placed the front end of the OLYMPUS260 electronic gastroscope above the anastomotic stenosis and pushed the guide wire of about 10 cm to the distal end of the anastomosis, and after fixing, gastroscope was withdrawn. Then, we selected a suitable size guide wire to insert into the anastomosis, and by using a dilator expansion, we inserted a stent pusher along the guide wire, then implanted the metal-membrane stent into the stenosis, and withdrew the stent pusher and guide wire. We re-inserted the gastroscope, observed the anastomosis, and then confirmed that there was no stent displacement, perforation, or bleeding. After that, the gastroscope was withdrawn. The patients were kept in a fasting state for 12 hours after the operation, and the eating time was determined according to the recovery situation.

### 2.6. Efficacy Evaluation

Degree of dysphagia (Stooler grade) and total response rate were assessed after treatment using the following indicators: significant efficiency + effective efficiency = total effective efficiency; markedly effective [9]: lumen diameter >1.2 cm, and symptoms such as dysphagia disappeared; effective: the lumen diameter was 0.6–1.0 cm, and symptoms such as dysphagia were improved; invalid: the above criteria were not met. As per the Stooler classification [10], the patients were classified as follows: grade I: occasional dysphagia, can eat all kinds of food, grade 0: no dysphagia, can eat all kinds of food, grade II: semi-liquid diet, and grade III: only liquid diet.

### 2.7. Statistical Processing

SPSS 20.0 statistical software was used for processing, and the count data were expressed as (%) and tested by *χ*^2^. The measurement data were represented by ($\bar{x}\pm s$), and the *t*-test was performed. Binary logistic regression analysis was used to analyze the independent factors leading to benign anastomotic stenosis in patients after operation, and finally, a prediction model was obtained. AUC was used to evaluate the accuracy of the model, and the Bootstrap method was used for internal verification to draw a calibration chart. *P* < 0.05 was considered statistically significant.

## 3. Results

### 3.1. Comparative General Information

Univariate analysis showed that age, gender, anastomosis method, tumor diameter, pathological type, past medical history, TNM staging, and expansion method did not affect postoperative benign anastomotic stenosis (*P* > 0.05) but affected anastomotic location and local blood supply. Eating time, however, will affect the occurrence of benign anastomotic stenosis (*P* < 0.05), as shown in Table 1.

### 3.2. Binary Logistic Regression

In binary logistic regression analysis, “whether benign anastomotic stenosis occurs after operation” was taken as the dependent variable, (assignment: benign anastomotic stenosis occurs =0 , no benign anastomotic stenosis occurs = 1 ). “anastomotic position (above tracheal bifurcatio =0 ; below tracheal bifurcation = 1), local blood supply (good = 0; poor = 1), and eating time (12h ≥ 0, 12h ≤ 1)“ was taken as independent variables.

The anastomotic stoma located above the tracheal bifurcation, poor local blood supply, and eating time ≥12 hours were independent factors leading to benign anastomotic stenosis after surgery (*P* < 0.05), as shown in Table 2.

### 3.3. Prediction Accuracy

In order to judge the quality of model fitting, it is necessary to use the model to predict the accuracy. The results show that the overall prediction accuracy of the model is 81.5%, and the model fitting is acceptable as shown in Table 3.

### 3.4. Validating the Prediction Model

The model is internally verified by the Bootstrap method, and the number of self-sampling is *B* = 1000, as shown in Table 4. At the same time, according to the selected independent influencing factors, a prediction model was obtained, namely, Logit (*P*) = 2.254 × anastomotic position + 1.818 × retention mode + 2.376 × feeding time.

The AUC is used to evaluate the simulation discrimination, where the AUC is 0.739 and the 95% CI is 0.636–0.841, as shown in Figure 1. This model has good accuracy and can better predict the occurrence of benign anastomotic stenosis in patients.

### 3.5. Analysis of Treatment Effect

In 55 cases with stenosis, after surgery, 23 cases (41.82%) were markedly effective, 29 cases (52.73%) were effective, 3 cases (5.45%) were ineffective, and the total effective rate was 94.54% (52/55%), of which Stooler 0 32 cases (58.18%) were grade I, 20 cases (36.36%) were grade I, and 3 cases (5.45%) were grade II, with a complication rate of 9.09% (5/55).

## 4. Discussion

Esophageal cancer is a high-incidence disease in the country. Currently, esophageal cancer is mainly treated by surgery, and although the effect is significant, complications such as postoperative anastomotic stenosis have always been a clinical problem [11]. Through investigation, it was found that 4 weeks after operation was a period of high incidence of anastomotic stenosis, 15% of patients were found to have anastomotic stenosis by endoscopy, and 42% of patients had swallowing function [12]. If effective measures are not taken to prevent it and the already-occurring anastomotic stenosis is not treated in time, the disease can seriously affect the postoperative nutritional status, daily life, and postoperative recovery. Based on this, it is necessary to focus on exploring the reasons for the occurrence of benign anastomotic stenosis after surgery, in order to provide a basis for the improvement of the surgical plan and the selection of preoperative indications in the future [13].

Binary Logistic regression analysis showed that eating time ≥12 hours, poor local blood supply, and anastomotic stoma located above the tracheal bifurcation were independent factors leading to benign anastomotic stenosis after surgery. The factors leading to benign anastomotic stenosis after surgery are as follows: ①Eating time: early eating can reduce the occurrence of anastomotic stenosis. This statement was also corroborated by this study. The results showed that eating time is an independent influencing factor. Earlier eating indicated a lower probability of occurrence. It is because early eating can produce mechanical stimulation and expansion, thereby reducing the occurrence of benign anastomotic stenosis. In this regard, it is necessary to eat within 12 hours, to reduce bleeding and oozing, promote gastrointestinal motility, reduce gastric acid reflux stimulation, and reduce the occurrence of stenosis. At the same time, it is necessary to pay attention to the actual situation of the patient and choose a reasonable eating time [14, 15]. ②Blood supply: univariate analysis showed that patients with poor blood supply had a higher probability of benign anastomotic stenosis because the reduction of oxygen supply to the local tissue of the anastomosis would promote hypercapnia and local anaerobic metabolism and stimulate connective tissue hyperplasia. Reducing the accumulation of acidic products and pH value will lead to a decrease in the healing ability and affect tissue self-repair, thereby increasing the incidence of benign anastomotic stenosis. In this regard, clinical attention should be paid to the preoperative and postoperative blood supply of patients and timely correction of the abnormal situation [16, 17]. ③Anastomotic location: studies have shown that the risk of stenosis varies in different anastomotic locations [18]. The higher the location, the easier and more stubborn it is for anastomotic stenosis to occur. The univariate analysis showed that the anastomotic stoma located above the tracheal bifurcation had a higher probability of stenosis, which may be because the blood supply of the high anastomotic stoma is very different from the gastric fundus and cardia, the blood supply above the tracheal bifurcation is poor, and it is vulnerable to mechanical traction. Due to the influence of tension, the proliferation of fibrous connective tissue is more obvious and the rate of anastomotic stenosis is higher. Therefore, for patients with high anastomotic stoma, it is necessary to choose a wide-diameter and large-sized stapler as much as possible to avoid stenosis [19].

Endoscopic dilatation is a common solution for the treatment of anastomotic stenosis after esophageal cancer surgery. It has the advantages of simple operation, minimal invasiveness, and safety. It can loosen the fibrous scar around the stenosis by an external force, break the muscle fibers at the anastomotic stenosis, and expand it. The esophageal lumen can improve the current symptoms such as dysphagia and eating obstruction [20]. However, with the deepening of stent implantation, it gradually replaced dilatation and became the preferred method, which can not only achieve the effect of dilation but can also reduce the number of expansions, relieve clinical symptoms, and improve postoperative quality of life [21]. Analysis of the results of this study showed that the total effective rate was 94.54%, only 3 cases had Stooler II and 5 cases had complications, indicating that stent implantation can effectively relieve symptoms such as swallowing dysfunction, and the treatment effect is significant and the safety is high. Analysis of the reasons showed that stent implantation can release the tear of fibrous scar tissue and expand the lumen, thereby relaxing and relieving esophageal anastomotic stenosis, and it can be assisted under endoscopy to better ensure clear vision, accurate positioning, safety, reliability, higher success rate, and prevention of complications

In conclusion, the reasons for the occurrence of benign anastomotic stenosis after operation are the feeding time, blood supply, and anastomotic location. Risk factors should be dealt within time, so as to reduce the postoperative stenosis rate and strengthen stent implantation. It can better improve postoperative symptoms such as dysphagia, and it has high safety and is worthy of promotion.

## Figures and Tables

**Figure 1:** ROC curve for validating the predictive model.

**Table 1:** Comparison of the general information of the two groups.

Indexes	Classification	Stenosis group (*n* = 55)	Nonstenosis group (*n* = 37)	*χ* ^2^ value	*P* value
Age	＜60 year	33 (60.00)	23 (62.16)	0.043	0.835
	≥60 year	22 (40.00)	14 (37.84)		
Gender	Male	31 (56.36)	20 (54.05)	0.048	0.827
	Female	24 (43.64)	17 (45.95)		
Tumor diameter	≤2 cm	35 (63.64)	25 (67.57)	0.151	0.698
	＞2 cm	20 (36.36)	12 (32.43)		
Anastomosis method	By stapler	38 (69.09)	26 (70.27)	0.015	0.904
	By manual anastomosis	17 (30.91)	11 (29.73)		
TNM phase	I∼II phase	19 (34.55)	13 (35.14)	0.003	0.954
	III∼IV phase	36 (65.45)	24 (64.86)		
Pathological type	Squamous cell carcinoma	44 (80.00)	30 (81.08)	0.016	0.898
	Nonsquamous cell carcinoma	11 (20.00)	7 (18.92)		
Anastomotic location	Above the tracheal bifurcation	30 (54.55)	9 (24.32)	8.272	0.004
	Below the tracheal bifurcation	25 (45.45)	28 (75.68)		
Medical history	Yes	10 (18.18)	6 (16.22)	0.059	0.807
	No	45 (81.82)	31 (83.78)		
Local blood supply	Well	16 (29.09)	25 (67.57)	13.255	＜0.001
	Not well	39 (70.91)	12 (32.43)		
Expansion method	By balloon	27 (49.09)	20 (54.05)	0.218	0.641
	By rod	28 (50.91)	17 (45.95)		
Eating time	＜12 h	16 (29.09)	24 (64.86)	11.519	0.001
	≥12 h	39 (70.91)	13 (35.14)		

**Table 2:** Factors leading to postoperative benign anastomotic stricture in patients.

Indexes	*B*	SE	Wald	Degrees of freedom	Significant	OR	95% CI	
							Lower limit	Upper limit
Anastomotic location	2.254	0.661	11.615	1	0.001	9.529	2.606	34.844
Local blood supply	1.818	0.554	10.777	1	0.001	6.158	2.080	18.227
Eating time	2.376	0.648	13.454	1	0.000	10.763	3.024	38.314
Constants	−5.954	1.357	19.247	1	0.000	0.003	—	—

**Table 3:** Summary of prediction accuracy of binary Logit regression.

—		Predictive value		Prediction accuracy
					0	1
True value	0	45	10	81.8%
	1	7	30	81.1%
Pool				81.5%

**Table 4:** Variables in the equation bootstrap.

Indexes	*B*	Bootstrap^a^				
		Deviation	Standard error	*P*	95% confidence interval	
					Lower limit	Upper limit
Anastomotic location	2.254	0.562	2.889	0.002	1.086	5.192
Local blood supply	1.818	0.127	0.665	0.002	0.814	3.430
Eating time	2.376	0.563	2.870	0.002	1.205	4.877
Constants	−5.954	−1.219	5.882	0.002	−12.366	−3.606

## Data Availability

The raw data supporting the conclusion of this article will be made available by the authors without undue reservation.
